# A DEA-Based Complexity of Needs Approach for Hospital Beds Evacuation during the COVID-19 Outbreak

**DOI:** 10.1155/2020/8857553

**Published:** 2020-09-30

**Authors:** Thyago C. C. Nepomuceno, Wilka M. N. Silva, Késsia T. C. Nepomuceno, Isloana K. F. Barros

**Affiliations:** ^1^Sapienza University of Rome, Dipartimento Di Ingegneria Informatica Automatica e Gestionale “Antonio Ruberti”, Via Ariosto, 25, Roma 00185, Italy; ^2^Federal University of Pernambuco, Núcleo De Tecnologia, Av. Marielle Franco, s/n-Km 59–Nova Caruaru, Recife, Brazil; ^3^Federal University of Pernambuco, Departamento De Bioquímica, Avenida Prof. Moraes Rego, s/n-Cidade Universitária, CEP: 50.670-420-Recife/PE, Recife, Brazil; ^4^Federal University of Pernambuco, Centro De Informática, Av. J. Anibal Fernandes, s/n, Cidade Universitária, CEP: 50.740-560-Recife/PE, Recife, Brazil

## Abstract

Data envelopment analysis (DEA) is a powerful nonparametric engineering tool for estimating technical efficiency and production capacity of service units. Assuming an equally proportional change in the output/input ratio, we can estimate how many additional medical resource health service units would be required if the number of hospitalizations was expected to increase during an epidemic outbreak. This assessment proposes a two-step methodology for hospital beds vacancy and reallocation during the COVID-19 pandemic. The framework determines the production capacity of hospitals through data envelopment analysis and incorporates the complexity of needs in two categories for the reallocation of beds throughout the medical specialties. As a result, we have a set of inefficient healthcare units presenting less complex bed slacks to be reduced, that is, to be allocated for patients presenting with more severe conditions. The first results in this work, in collaboration with state and municipal administrations in Brazil, report 3772 beds feasible to be evacuated by 64% of the analyzed health units, of which more than 82% are moderate complexity evacuations. The proposed assessment and methodology can provide a direction for governments and policymakers to develop strategies based on a robust quantitative production capacity measure.

## 1. Introduction

The past months scourged the world with a novel coronavirus identified as the cause of a pneumonia outbreak first detected in Wuhan, province of Hubei, China. The severe acute respiratory syndrome coronavirus-2 (SARS-CoV-2) is responsible for a declared worldwide pandemic having more than a million confirmed cases and dozens of thousands of deaths, keeping a quick spread [1, 2]. The prompt virus outbreak causes a much bigger problem than lethality: a large number of infected patients require hospitalization and intensive care due to complications worsening the clinical condition. When several patients need such intensive care at the same time, the hospitals and other health service units with limited resources end up overloaded. As a result, the health systems collapse due to the unavailability of beds, ventilators, and technical resources for new hospital admissions, fatigue, and overloading health teams. Thus, hospital beds acquisition and evacuation are crucial to increase the response capacity to face the crisis [3].

Data envelopment analysis is a powerful nonparametric mathematical programming tool for the technical efficiency estimation of many service units in different economic activities, such as financial institutions and educational and health systems [4–7]. Hospitals are a wide source of efficiency assessments. Some of the most relevant results provide the potential for health improvement based on the expansion of results (e.g., hospitalizations, patient recoveries, performed surgeries, medical prescriptions, among others) or based on the contraction of resources (e.g., nurses, assistants, physicians, infected patients (nondiscretionary), beds, equipment, among others). Such prospects are possible through the envelopment of data, which estimates the industry's efficient production capacity.

This study introduces a novel application to provide an optimal number of hospital beds technically feasible to be evacuated and allocated for urgent hospitalizations through best practices, applicable during the COVID-19 crisis. The methodology is based on the Brazilian Healthy Complexity of Needs prioritization and can be extended to any health system with a similar or different classification of disease and medical specialties.

## 2. Literature

The increasing pressure on limited resources of health systems during the pandemic has highlighted the need for efficiency-based tools and methodologies to offer new combined perspectives on how to use the hospital's facilities, resources, and capabilities optimally. Ordu et al. [8, 9] develop an interesting decision support tool for modelling capacity constraints, and allocating hospitals' resources, combining discrete event simulation and forecasting techniques. The application in the accident and emergency department captures the outpatient demand for each specialty by age and first/followup referrals and the entire service pathway on different scenarios. Similar approaches aiming at providing increased operational efficiency and high-quality patient care are claimed to offer a considerable improvement in the hospitals' capacity response and average patient length of stay [10, 11]. A measure for the required number of optimal emergency beds, however, is a limitation acknowledged by the authors in these and other operations approach.

The nonparametric frontier estimations of data envelopment analysis can aid managers and policymakers in attaining such a prospect. The weight optimization based on pairwise evaluations scales the used resources and generated products of each service unit, providing a robust measure for the technical efficiency, which can be adapted for inverse output/input relations [12], exogenous or nondiscretionary resources [13–15], and time-series self-evaluations [16–18]. As a result, an estimation for the optimal production capacity for any size service unit is available for decision-making. In the case of hospitalizations, this optimal capacity measure can be translated into an efficient number of hospital beds, equipment, costs, or human resources required for the production of health using internments (hospitalizations) as a proxy for this product.

This instrument, besides offering a relative measure for hospitals' technical efficiency based on the maximum, yet feasible, production configuration, can determine peers of efficiency for benchmarking performance metrics and identifying opportunities for improvement and support resource allocation schemas based on production slacks. Many assessments of health efficiency follow this avenue, for instance, the recommendations of Kounetas and Papathanassopoulos [19] regarding the efficiency of Greek hospitals and Zare et al. [20] using a hybrid data envelopment analysis and game theory methodology for performance measurement in health service units. This interesting perspective of frontier estimations can provide the optimal number of resources to be (re-) allocated from inefficient units through best practices during epidemic crises.

The most common variables considered in modelling the production technology of health systems are the number of beds for hospitalizations, personal protective equipment (PPE) and other technical equipment, drugs, human capital (physicians, nurses, unlicensed assistants, and other staff), hospital infrastructure, costs of service (in many categories), and funding as inputs, and medical prescriptions, number of hospitalizations, outpatient procedures, inverse mortality rate, patients discharged, number of surgeries, and testing as outputs [6,19–26]. Nevertheless, different combinations of output/input can be used in assessments of hospitals' performance, depending on the problem statement and purpose. For instance, Hadad et al. [21] show an interesting nonconventional evaluation which resorts to life expectancy and infant survival rate as the parameters for the health product in two efficiency models, considering the physicians' density, inpatient bed density, expenditures, gross domestic product (GDP), and fruit and vegetable consumption, adding a different perspective in the efficiency assessment.

Most hospitals, in general, during the last weeks, and especially intensive care units (ICUs) and emergency departments (EDs) are constantly required to cope with a recurrent daily-based crisis ignited by the novel coronavirus outbreak. Gul & Guneri [27] and Gul et al. [28] discuss the importance of these sectors, dedicated to patients in need of urgent and commonly complex care, in a comprehensive review of literature and evaluation. In addition to the impact on these sectors, the pandemic has affected other specialties that are not directly related to the treatment of respiratory syndromes, where the resource becomes committed in order to prevent the collapse of an entire health system. In most assessments, different conditions and specialties are taken into consideration in several hospital departments, which brings a real contribution of hybrid models to the strategic planning of health service units.

The different specialties carried out by health service units are subject to different and varied heterogeneous factors that are connected to institutional arrangements, population characteristics, location, and socioeconomic or environmental determinants. The linear programming scales the differences through the output/input ratio of each health unit by comparing small units with a benchmark in the efficiency frontier presenting similar input-to-output configuration. Nevertheless, such heterogeneity has a considerable subjective value in the decision maker's perspective, which, despite the objective programming techniques, requires value judgments and preference elicitations on different decision criteria. Multiple criteria methodologies, for instance, Pergher & Vaccaro [29] outranking model based on the Electre Tri, Mendonça et al. [30], grey theory approach for risk assessments, and many others [31–36], can be relevant adapting on this prospect.

## 3. Methodology

The technical efficiency is traditionally understood as a ratio between the generated outputs and used inputs of a production process. Charnes et al. [37] and Banker et al. [38] through a mathematical linear dual formulation for multiple outputs/inputs configurations in the efficiency problem introduced the so-called data envelopment analysis (DEA). Today, this is the most common approach to assess the efficiency and productivity of many decision-making units (DMUs) in the number of surveys, applications, methodologies, and computational developments [39, 40]. The mathematical programming provides, among other results, the optimal amount of resources to save or products to increase so that an inefficient service unit becomes efficient.

The multidimensional production structure of hospitals and healthcare centres, however, requires a meticulous approach to define which resources need to be reduced in order to improve the health results. According to Lin & Kuo [41], different patient's complexity relies on different health service providers for different clinical specialties, which may jeopardize the slack reduction consistency in the technical efficiency analysis because potential performance improvements in hospitalizations by equally reducing the hospital beds, for instance, for all specialties, may be neither feasible nor coherent for each particular hospital context. An interesting solution is suggested by Ferreira and Marques [42]. According to this study, there is no need for complexity adjustment if one accounts for the operational environment surrounding the hospital. Conditional frontier analysis [15, 43] can add an interesting perspective by considering those environmental determinants in the frontier estimation.

An alternative avenue through a two-step methodology is proposed in this assessment. Estimations for the beds' evacuation is proposed by prioritizing the slack reduction according to the complexity of needs on the most common medical specialties to provide support for bed reallocations during an epidemic crisis. The first step consists of applying nonparametric frontier estimations for the full production capacity of the health service units (the maximum feasible production configuration for each hospital) based on hospital admissions as the main output and hospital beds as one of the many discretionary resources. Similar to many assessments of health systems efficiency, the number of beds is considered a proxy for hospital capital [31–36, 44]. That way, depending on the scale of operations and keeping everything else constant, the lower the usage of this resource, the higher the efficiency for the health service unit. Following similar resource optimization approaches [45, 46], the objective in this assessment is to provide an optimal number of beds to be evacuated and allocated for potential COVID-19 cases, instead of reduction.

For the second step, the optimal number of beds to be reallocated (based on best practices) are prioritized according to the complexity of needs for each medical specialty. The complexity of needs in the Brazilian Health System is the degree of complexity each health problem presents and the requirement for specialized knowledge. There are three categories: basic care, moderate complexity, and high complexity. Each category is defined in Table 1.

Hospitalizations have moderate (*ε*_low_) or high (*ε*_high_) complexity of needs admissions. Consider a set of *j*=1,2,3,…, *m* health service units using *x*_*i*_|*i*=1,2,3,…, *n* hospital inputs to produce *y*_*r*_|*r*=1,2,3,…, *s* outputs. Consider “*o*” the service unit under evaluation and “*ε*,” the sum of both moderate and high complexity of needs hospitalizations, a proxy for the prioritization of beds evacuation. The optimal feasible contraction (evacuations) of high complexity hospitalization beds is as follows:

(1) $$\begin{array}{c} Ev_{A+}=\left\{\begin{array}{cc} \varepsilon \left(1-\theta^{*}\right)-\varepsilon_{\mathrm{low}}, & \mathrm{when}\varepsilon \left(1-\theta^{*}\right)-Ev_{A-}>0,\\ \mathrm{0,} & \mathrm{Otherwise}. \end{array}\right. \end{array}$$

The optimal feasible contraction (evacuations) of moderate complexity beds is as follows:

(2) $$\begin{array}{c} Ev_{A-}=\left\{\begin{array}{cc} \varepsilon_{\mathrm{low}}, & \mathrm{when}\varepsilon \left(1-\theta^{*}\right)-\varepsilon_{\mathrm{low}}\geq 0,\\ \mathrm{0,} & \mathrm{Otherwise,} \end{array}\right. \end{array}$$

where *θ*^*∗*^=min(*θ*)|(∑_*j*=1_^*m*^*z*_*j*_*x*_*ji*_ ≤ *θx*_*oi*_; ∑_*j*=1_^*m*^*z*_*j*_*y*_*jr*_ ≥ *y*_*or*_; ∑_*j*=1_^*m*^*z*_*j*_=1&*z*_*j*_ ≥ 0) is the efficiency score for the production technology under variable returns to scale [9, 14].

Equations (1) and (2) state that the optimal number for beds evacuation of high complexity admissions depends on the number of evacuated beds of moderate complexity. In other words, the optimal number for beds evacuation of high complexity hospitalizations is the remaining feasible contraction of beds after all moderate complexity admissions are evacuated. As an example, considering an efficiency score *θ*^*∗*^  = 0.8, the service unit may improve efficiency by producing the same result using (1–0.8) = 20% fewer resources. Considering 100 hospital beds allocated to admissions of both low and high complexity of needs as the discretionary input |*ε*_low_ = 15 and *ε*_high_ = 85, the number of beds to be evacuated having moderate complexity is *Ev*_*A*−_ =*ε*_low_=15 beds and the number of beds to be evacuated having high complexity is the remaining *Ev*_*A*+_ =*ε*(1 − *θ*) − *ε*_low_=20 − 15=5 beds.

Adding (1) and (2) into the DEA formulation, we can infer the optimal number for beds evacuation (*Ev*_*A*_) based on the complexity of needs prioritization:

(3) $$\begin{array}{c} Ev_{A}\left(\mathrm{x,y,\varepsilon}\right)\;=\left\{\begin{array}{cc} Ev_{A-}=\varepsilon \left[1-\min\left(\theta \right)\left|\begin{array}{c} \overset{m}{\underset{j=1}{\sum }}z_{j}x_{ji}\leq \theta x_{oi},\;\forall i=1,2,\ldots ,n\\ \overset{m}{\underset{j=1}{\sum }}z_{j}y_{jr}\geq y_{or},\;\forall r=1,2,\ldots ,s\\ \overset{m}{\underset{j=1}{\sum }}z_{j}=1,z_{j}\geq 0,\;\forall j=1,2,\ldots ,m \end{array}\right.\right], & \text{when }\varepsilon \left(1-\theta^{*}\right)-\varepsilon_{\mathrm{low}}\leq 0,\\ Ev_{A+}+Ev_{A-}=\left(\varepsilon \right)\left[1-\min\left(\theta \right)\left|\begin{array}{c} \overset{m}{\underset{j=1}{\sum }}z_{j}x_{ji}\leq \theta x_{oi},\;\forall i=1,\ldots ,n\\ \overset{m}{\underset{j=1}{\sum }}z_{j}y_{jr}\geq y_{or},\;\forall r=1,\ldots ,s\\ \overset{m}{\underset{j=1}{\sum }}z_{j}=1,z_{j}\geq 0,\;\forall j=1,\ldots ,m \end{array}\right.\right]-\varepsilon_{\mathrm{low}}+Ev_{A-}, & \mathrm{Otherwise}. \end{array}\right. \end{array}$$

Full concepts and definitions concerning the complexity of needs assistance in the Brazilian Health System and a list with the related medical specialties are available in [47].

## 4. Data

In the first step of the evaluation, an input-oriented variable returns to scale model is conducted. Pernambuco's State Secretariat for Budgeting and Planning (SEPLAG) provided data regarding 373 from the 1136 health services units in the state. For this assessment, we have selected the 88 most important hospitals and healthcare centres based on the volume of hospitalizations. Due to data limitations, the number of doctors, surgeons, and general physicians is not considered in the analysis. For most medical specialties, ward rounds for inpatient care by physicians occur once a day or after a week, depending on the patient treatment plan or condition. This context let us assume that the inclusion or removal of these professionals may not shift the efficiency prospects compared to nurses and other health staff which are in direct contact with hospitalizations. The inputs are the number of nurses, nursing assistants, and licensed healthcare technicians and the cost of hospitalizations and the sum of hospital beds for three categories (specialties): medical clinics (comprehensive care for individuals aging over 12 years, in critical or semicritical conditions, and who do not need surgical treatment), surgical clinics (reserved for preoperative and postoperative care), and obstetrics. The output is the number of hospital internments (hospitalizations).

Table 2 and Figure 1 report the main descriptive statistics. Costs refer only to hospitalizations expenditure considering the three specialties. On average, R$ 8,073,821 (about US$ 1.5 million) is spent per health unit in hospitalizations for a typical year. Nursing assistants and nursing technicians are two professional categories working in outpatient sectors usually performing basic care planned by the nurse, such as administration of medicines, vaccines, dressings, performing patient hygiene, and sterilization of medical equipment. Due to the similarity of both categories, they were aggregated into one input named “assistants and technicians”.

In general, the 88 most important health units in the state sums 16336 of those professionals, 5452 nurses, and 12388 beds, spent more than R$ 710 million (about US$ 132 million) in one year, and were responsible for 462175 hospitalizations and 5252 hospitalizations per unit on average. This means 0.07% (88 hospitals) were responsible for 27.02% of all hospitalizations in the state. Figure 1 illustrates the descriptive statistics in boxplots visualizations. Most of the outliers are public hospitals characterized by a high demand for health services.

## 5. Results and Discussion

Tables 3 and 4 summarize the main results. We have 26 hospitals working at full capacity in the state, serving as peers (benchmarks) for the remaining inefficient health units. These units are producing the maximum possible admissions a hospital can produce during a year given the current production technology, equipment, and human resource. It is worth mentioning that, for some of the ranked hospitals, the efficiency comes at the cost of quality due to the high demand for health services and overcrowded public hospitals. The total of 3772 beds are feasible to be evacuated and reallocated for new COVID-19 cases in one year considering the remaining inefficient units formalization of new service protocols, postponing surgeries and decreasing the patient length of stay in hospitals through best practices from the peers, of which 2883 are related to moderate hospitalizations and 889 high complex cases.  Table 4 has the remaining hospitals and their potential for bed evacuation during the crisis.

Figure 2 illustrates the overall production capacity with the efficiency frontier estimation by the envelopment of data under a variable returns to scale technology. In the visualization of Figure 2, the inputs in the *x* label are aggregated by simple summing with no specific weight for this aggregation. One should be alerted that a multiple-input to one output plot may not necessarily place the multiefficient health service units on the two-dimensional frontier, serving only illustration purposes. The traditional radial variable returns to scale model can be the most interesting option for the objective of incorporating the complexity of needs in a second step defining the feasible options for resource evacuation among the specialties. Because of the characteristic of data (beds available by medical specialties), we can prioritize the reduction of beds (and related resources uniformly) according to the complexity of their specialty. The points on the frontier represent the efficient hospitals reported in Table 3, which are benchmarks for best practices. The remaining inefficient units (under the frontier) in this illustration become efficient either by producing more hospitalizations with the same level of used inputs or by reducing the used inputs keeping hospitalizations at the same level or by a combination of both. In the input-oriented model of this assessment, efficiency is obtained by reducing (and reallocating) the number of beds keeping the same amount of hospitalization. This can be possible by applying some of the benchmark strategies for reducing the length of stay. In this representation, the most inefficient unit (the most distant point from the frontier) is one of the most important private hospitals in the state, having a considerable number of available beds for reallocation in a typical year.

Table 5 reports the main prospects for the assessment. The evacuation of hospital beds are prioritized according to the complexity of needs for the many medical specialties each health service units operate. The monthly estimates are evacuation projections based on the efficient production capacity of hospitals, which can be used during the pandemic critical months. Twenty-three out of the 57 health service units with potential for bed evacuations do not require high complexity evacuations. Twenty out of the 57 require less than 50% high complexity evacuations. This methodology helps the policymaker concentrate attention on the hospital with the best potential and less critical services to evacuate and reallocate beds and related resources through best practices referred from the benchmarking peers of the evaluation.

## 6. Conclusions

The assessment provided a framework for the application of nonparametric frontier methods of the DEA family to estimate the technically feasible capacity of hospitalizations, which, combined with prioritization methodologies for medical specialties such as the cmplexity of needs in Brazil, can disclose valuable support for policymakers to prevent an eventual collapse of health systems during the COVID-19 epidemic crisis. The methodology can be adapted to other localities, or decision criteria, providing a systematic approach for resource allocation through hospitals during the pandemic.

A valuable extension for the assessment of the health service units technical efficiency is the frontier estimation based on time-series production data instead of pairwise comparisons. Due to the many particular differences regarding the production technology of hospitals, an approach based on internal rather than industrial capacity can be more deductive and coherent.

Another interesting value can be added by the definition of beds' evacuation based on multiple decision criteria besides the complexity of needs. Important clinical aspects of hospital internments such as the gravity of diseases, flexibility for resource transfer among the medical specialties, and substitution potential can orientate decisions of managers and policymakers closer to each health unit reality. In addition, the usage of fuzzy data for the assessment of network system such as a hospital can aid valuable support [48]. This analysis can provide a direction for public administrations to perform some of their strategies based on an objective quantitative production capacity measure and support subjective decision-making with the inclusion of such aspects.

An extension of the current application investigating the efficiency evolution and the hospitalization efficacy against COVID-19 can be very useful for policymakers. A time-series evaluation, as suggested by Nepomuceno et al. [49], can be performed using time-series data regarding the period before and after the implementation of beds reallocation schema based on each specialty complexity of needs. The first results of this assessment were disclosed to state authorities, hoping to contribute to how to mitigate the drastic effects of the current crisis in the available resources.

## Figures and Tables

**Figure 1:** Boxplots visualization. ^*∗*^Hospitalization costs (expenditure) in 100000. ^*∗∗*^Number of hospitalizations in 100.

**Figure 2:** Efficiency frontier.

**Table 1:** Complexity of needs categories.

Basic care: the first level is characterized by a set of actions and practices using low-density technologies to solve health issues of greater frequency but low severity, including a list of simpler and cheaper procedures. The procedures in this category are capable of meeting most of the community's common health problems.

Moderate complexity: composed of actions and services aiming at meeting the main public health issues whose assistance in the clinical practice requires the availability of specialized professionals and the usage of technological resources for diagnostic, support, and treatment.

High complexity: common for more severe health issues; this category is characterized by a set of procedures involving high technology and high cost, aiming at providing access to highly specialized knowledge and qualified services.

**Table 2:** Variables and descriptive statistics.

Variables		Min.	1^st^ Qu.	Median	Mean	3^rd^ Qu.	Max.	Std. Dev.

Inputs	Assistants and technicians	4.0	27.5	75.5	185.6	212.2	1409.0	271.54
	Nurses	1.00	7.00	15.50	61.95	79.50	617.00	96.98
	Hospital beds	11.00	41.75	72.50	140.77	155.00	1075.00	181.54
	Costs	28388	225080	1804658	8073821	5137736	101663545	17038427

Output	Hospitalizations	74.0	527.8	2530.0	5252.0	7625.8	41678.0	7155.14

**Table 3:** Efficient hospitals at full capacity of admissions.

Health service units	Beds	Peering

IMIP	1075	N/A
Hospital Da Restauração	790	9 units
Hospital Otavio De Freitas	620	N/A
Hospital Getulio Vargas	545	2 units
Hospital Barao De Lucena	340	1 unit
Hospital Dom Malan	259	8 units
Hospital Miguel Arraes	173	4 units
Hospital Pelopidas Silveira	170	3 units
HMR Dra Merces P. Cunha	150	43 units
HM Santa Maria	146	7 units
HR Fernando Bezerra	98	3 units
CH Dr Jose E. De Moura	91	15 units
HMC C. S. Bom Jesus	70	18 units
IBVASF	67	4 units
HI Palmira Sales	62	19 units
Casa De Saúde São Jose	59	2 units
PM Pr. Barros Lima	57	7 units
Mat. Dr Luiz Leite	42	4 units
Hospital Ermirio Coutinho	41	11 units
HMM. Olimpio M G. Lins	26	20 units
UM Kyola	23	24 units
Hosp. Genezio F. Xavier	22	1 unit
UM Dr Jose M. Monteiro	16	15 units
UM Jose Dantas Filho	15	2 units
HM Alice Figueira	14	13 units
UM Maria Eliziaria Paes	11	5 units

**Table 4:** Hospitals with potential for bed evacuations.

DMU	Efficiency	Beds	Evacuations

1	0.078	744	686
2	0.586	425	176
3	0.268	191	140
4	0.427	234	134
5	0.619	255	97
6	0.511	197	96
7	0.277	128	92
8	0.352	142	92
9	0.812	407	76
10	0.668	210	70
11	0.653	198	69
12	0.675	193	63
13	0.561	138	61
14	0.664	180	61
15	0.566	130	56
16	0.875	426	53
17	0.601	125	50
18	0.686	150	47
19	0.543	81	37
20	0.685	115	36
21	0.619	90	34
22	0.668	96	32
23	0.408	52	31
24	0.662	82	28
25	0.535	52	24
26	0.615	61	23
27	0.690	74	23
28	0.772	98	22
29	0.605	56	22
30	0.499	44	22
31	0.629	59	22
32	0.670	59	19
33	0.643	54	19
34	0.692	60	18
35	0.655	51	18
36	0.666	50	17
37	0.874	130	16
38	0.59	39	16
39	0.697	46	14
40	0.810	71	13
41	0.893	108	12
42	0.933	173	12
43	0.723	38	11
44	0.896	111	11
45	0.925	148	11
46	0.745	37	9
47	0.892	88	9
48	0.691	24	7
49	0.886	61	7
50	0.844	32	5
51	0.979	244	5
52	0.810	21	4
53	0.840	26	4
54	0.895	32	3
55	0.920	42	3
56	0.898	20	2
57	0.902	20	2
58	0.966	39	1
59	0.974	35	1
60	0.979	31	1
61	0.987	61	1
62	0.978	22	0

**Table 5:** Potential for bed evacuations according to the complexity of needs.

DMU	Moderate complexity(%)	High complexity(%)	Monthlyestimate

1	100	83	57
2	94	0	15
3	100	67	12
4	60	0	11
5	58	0	8
6	68	0	8
7	100	51	8
8	100	57	8
9	55	0	6
10	70	0	6
11	65	0	6
12	100	4	5
13	100	7	5
14	100	31	5
15	0	43	5
16	39	0	4
17	100	26	4
18	51	0	4
19	100	28	3
20	100	18	3
21	100	28	3
22	100	12	3
23	100	51	3
24	100	32	2
25	100	27	2
26	100	29	2
27	100	12	2
28	86	0	2
29	100	31	2
30	100	0	2
31	100	24	2
32	100	19	2
33	100	17	2
34	100	47	2
35	100	18	1
36	100	12	1
37	23	0	1
38	100	30	1
39	100	24	1
40	43	0	1
41	2	0	1
42	9	0	1
43	16	0	1
44	16	0	1
45	100	3	1
46	100	1	1
47	49	0	1
48	100	5	1
49	100	3	1
50	0	10	1
51	21	0	1
52	68	0	1
53	24	0	1
54	9	0	1
55	26	0	1
56	38	0	1
57	16	0	1
58	88	0	1
59	100	8	1
60	78	0	1
61	100	17	1
62	53	0	1

## Data Availability

Readers can access the data related to the findings of this study upon request.
